The article "Silencing Cardiac Troponin I-Interacting Kinase Reduces Lipopolysaccharide-Induced Sepsis-Induced Myocardial Dysfunction in Rat by Regulating Apoptosis-Related Proteins" was published in 2021. Journal: Biomed Res Int.

# Silencing Cardiac Troponin I-Interacting Kinase Reduces Lipopolysaccharide-Induced Sepsis-Induced Myocardial Dysfunction in Rat by Regulating Apoptosis-Related Proteins

**DOI:** 10.1155/2021/5520051

**Published:** 2021-05-27

**Authors:** Dong Yang, Yanzhou Jiang, Haixia Qian, Xiaomin Liu, Liguo Mi

**Affiliations:** ^1^Department of Emergency (Xiangjiang Hospital), The Third Hospital of Hebei Medical University, Shijiazhuang 050051, China; ^2^Department of Orthopaedics, Weifang City Hanting People's Hospital, Weifang 261100, China; ^3^Department of Cardiovascular Medicine, Weifang City Hanting People's Hospital, Weifang 261100, China; ^4^Department of Anatomy, Hebei Medical University, Shijiazhuang 050017, China

## Abstract

The aim of this study was to investigate the effect of cardiac troponin I-interacting kinase (*TNNI3K*) on sepsis-induced myocardial dysfunction (SIMD) and further explore the underlying molecular mechanisms. In this study, a lipopolysaccharide- (LPS-) induced myocardial injury model was used. qRT-PCR was performed to detect the mRNA expression of *TNNI3K*. Western blot was conducted to quantitatively detect the expression of *TNNI3K* and apoptosis-related proteins (Bcl-2, Bax, and caspase-3). ELISA was performed to detect the content of lactate dehydrogenase (LDH) and creatine kinase (CK). TUNEL assay was used to detect the apoptosis of H9C2 cells. In LPS-induced H9C2 cells, *TNNI3K* was up regulated. Besides, the CK activity, the content of LDH, and the apoptosis of H9C2 cells were significantly increased after treatment with LPS. Silencing TNNI3K decreased the LDH release activity and CK activity and inhibited apoptosis of H9C2 cell. Further research illustrated that si-TNNI3K promoted the protein expression of Bcl-2 and decreased the protein expression of Bax and cleaved caspase-3. The study concluded that TNNI3K was upregulated in LPS-induced H9C2 cells. Importantly, functional research findings indicated that silencing TNNI3K alleviated LPS-induced H9C2 cell injury by regulating apoptosis-related proteins.

## 1. Introduction

Sepsis can lead to multiorgan dysfunction, among which sepsis-induced myocardial dysfunction (SIMD) is a serious complication [1]. The initial manifestation of SIMD is contractile systolic damage associated with compensatory diastolic ventricular dilatation. As the disease progresses, diastolic dysfunction occurs and diastolic compliance decreases, eventually leading to total heart failure [2]. A growing body of evidence suggests that myocardial dysfunction may exacerbate hemodynamic instability, which is a key cause of death and an independent risk factor for death in patients with sepsis [3]. Besides, two clinical studies have shown that patients with septic associated systolic dysfunction (sepsis induced cardiomyopathy) have an increased mortality rate of up to 80%, compared with patients with sepsis with normal systolic function [4, 5]. Currently, fluid resuscitation and contractile drugs such as dobutamine or levosimendan are the main strategies for the treatment of SIMD. However, fluid overload can be harmful to the heart, and the effectiveness of muscle contractile agents remains controversial [6, 7]. Therefore, it is urgent to explore new treatment methods for SIMD.

Despite years of research, the mechanism by which sepsis induces SIMD is complex and controversial [8]. At present, the main mechanisms leading to SIMD include cytokine action, mitochondrial dysfunction, release of induced nitric oxide, autonomic nervous dysfunction, calcium circulation disorder, and apoptosis of cardiomyocytes [9–12]. Among them, apoptosis of cardiomyocytes is an important factor in SIMD. In the apoptosis mechanism, the TNF-a receptor-mediated death pathway, mitochondria-dependent caspase activation pathway, and mitogen-activated protein kinase (MAPK) activation pathway are the three pathways to induce apoptosis of myocardial cells. Therefore, it is of great significance to further explore the molecular mechanism of SIMD and explore effective ways to prevent infectious cardiac dysfunction.

Cardiac troponin I interaction kinase (TNNI3K) is a member of the mitogen-activated protein kinase (MAPKKK) family and cardiac anchor protein repeat kinase (CARK), which was originally cloned by researchers of Peking University Union Medical College in 2003 [13]. TNNI3K is selectively expressed in cardiac tissue and is observed in fetal and adult hearts. Except for a small amount of expression in the brain and testis, TNNI3K is almost absent in other tissues [14]. Studies have shown that TNNI3K plays a vital role in important parts of cardiac biology and heart diseases, including viral myocarditis, cardiomyopathy, and cardiac conduction, indicating that TNNI3K is a promising target for the treatment of heart diseases [15–17]. However, there have been few studies on whether TNNI3K plays a role in the apoptosis of septic cardiomyocytes.

Herein, the aim of this study was to establish a rat model of sepsis treatment with LPS to investigate the effect of TNNI3K on SIMD.

## 2. Materials and Methods

### 2.1. Cell Culture

The rat myocardial cells (H9C2) were obtained from American Type Culture Collection (ATCC, Manassas, VA). After resuscitation, they were cultured in RPMI-1640 medium containing 10% fetal bovine serum (FBS, Beyotime, Beijing, China) in a humidified environment. When cells attained 70% to 80% confluences, transfection experiments could be conducted.

### 2.2. Experimental Groups

To establish a model of myocardial injury, H9C2 cells were divided into two groups: (1) control group, treatment with 10% FBS, and (2) LPS group, treatment with 10 *μ*g/mL LPS for 24 h. To detect the effect of TNNI3K on myocardial injury, the cells were divided into six groups: (1) control group, treatment with 10% FBS; (2) LPS group, treatment with 10 *μ*g/mL LPS for 24 h; (3) si-NC group, cotransfection with si-NC; (4) si-NC+LPS group, cotransfection with si-NC and LPS; (5) si-TNNI3K, cotransfection with si-TNNI3K; and (6) si-TNNI3K+LPS group, cotransfection with si-TNNI3K and LPS. This study was approved by the Ethics Committee of the Third Hospital of Hebei Medical University.

### 2.3. Cell Transfection

si-NC and si-TNNI3K were constructed by Ribobio Corporation (Guangzhou, China), and plasmid dosage per transfection was 100 ng. The cells were divided into groups according to the experimental plan and inoculated into 6-well plates. Lentivirus infection was carried out after the cells adhered to the wall. After 24 h, 10 *μ*g/mL LPS cells were added for 24 h.

### 2.4. Quantitative Real-Time PCR

TRIpure reagent (Invitrogen, USA) was used to isolate the total RNA from samples, and PrimeScript RT kit (TaKaRa, Otsu, Japan) was used for reverse transcription. After the sample was prepared, the expression level was detected with SYBR green, and GAPDH was controlled as the internal parameter. 2^-*ΔΔ*Ct^ methods represented the fold changes of gene expression. The primer sequences for this experiment are shown below: TNNI3K sense (CGATACCGAGCCAACACCTA) and antisense (GCACCCACAAACTGAACCAC) and *β*-actin sense (GGAGATTACTGCCCTGGCTCCTAGC) and antisense (TGGCCGGACTCATCGTACTCCTGCTT).

### 2.5. Western Blot Analysis

According to the manufacturer's instruction, the proteins were extracted and its concentration was measured. Subsequently, the prepared protein was separated by polyacrylamide-SDS gels and then transferred onto PVDF membranes (Roche, Switzerland). After blocking, the PVDF membrane was subjected to incubation with primary antibodies: TNNI3K (1 : 1000, Abcam), Bcl-2, Bax, and cleaved caspased-3 (1 : 500, Wanleibio, Wuhan, China). On the following day, the membrane was incubated with the secondary antibody at 37°C for 45 min and the intensity of protein expression was detected by ECL chemiluminescence (Beyotime, Beijing, China).

### 2.6. Measurement of Creatine Kinase (CK) by ELISA

Concentrations of CK in the LPS-induced H9C2 cells were assessed by ELISA using a commercially available ELISA kit (USCN Business Co., Ltd., Wuhan, China) according to the manufacturer's instructions.

### 2.7. Lactate Dehydrogenase (LDH) Assay

Briefly, cells (1 × 10^4^) were seeded into 96-well plates and cultured for 12 h. After being collected, the LDH release activity from damaged cells was measured using a Cytoxicity Detection Kit (Roche, Basel, Switzerland). The absorbance values at 490 nm were detected using a microplate reader (Bio-Rad).

### 2.8. TUNEL Assay

TUNEL detection kit (Beyotime, Beijing, China) was used to detect the apoptosis of H9C2 cells. First, myocardial cells were fixed with 4% formaldehyde and then washed in PBS containing proteinase K (20 *μ*g/mL) at 37°C. Afterwards, H9C2 cells were incubated overnight with the two (1 and 2, 1 : 10) TUNEL reagents. Finally, TUNEL staining was observed under an optical microscope (Olympus, Tokyo, Japan).

### 2.9. Statistical Analysis

All the data were analyzed by Statistical Package for Social Sciences19.0 (SPSS, Chicago, IL, USA). One-way ANOVA followed by Dunnett's multiple comparison was applied to assess the differences between the groups. *P* < 0.05 indicated a significant difference between groups.

## 3. Results

### 3.1. TNNI3K Was Highly Expressed in LPS-Induced H9C2 Cells

To investigate the role of TNNI3K in myocardial injury in rats, we measured the expression of TNNI3K at both transcriptional and translational levels. As indicated in Figure 1(a), the mRNA level of TNNI3K was sharply upregulated as comparison to control group (*P* < 0.01). Similarly, in the translational level, LPS-induced H9C2 cells also showed a significant increase protein expression of TNNI3K (Figure 1(b)). Correspondingly, the average OD value was evidently increased in the LPS group (Figure 1(c), *P* < 0.01).

### 3.2. LPS-Induced Myocardial Injury

As presented in Figure 2(a), the activity of CK was significantly increased in the LPS group when compared with the control group, indicating LPS-induced myocardial injury (*P* < 0.01). To further verify this conclusion, LDH assay and TUNEL assay were conducted to detect the death status and apoptosis of the cells. In LDH assay, we found that the LDH release activity from H9C2 cells was remarkably increased, suggesting that LPS aggravated H9C2 cell injury (*P* < 0.01, Figure 2(b)). In TUNEL assay, the fluorescence activity of LPS-induced H9C2 cells was significantly enhanced. Correspondingly, the mean fluorescence intensity of the LPS group also increased significantly (*P* < 0.01, Figures 2(c) and 2(d)).

### 3.3. Silencing TNNI3K Alleviated LPS-Induced H9C2 Cell Injury

To further explore the effect of TNNI3K in myocardial injury in rats, we knock down TNNI3K in H9C2 cells. As shown in Figure 3(a), in the i-TNNI3K group, the protein level of TNNI3K was significantly reduced. Consistently, the average of the OD value in the si-TNNI3K group was also significantly reduced after transfection with si-TNNI3K (*P* < 0.01, Figure 3(b)), and a high knockout efficiency si-TNNI3K-1 was selected for subsequent research. In ELISA assay, CK activity increased significantly after treatment with LPS. However, when TNNI3K was knocked out, the CK activity decreased remarkably, with the si-TNNI3K-1 group having the most significant change (*P* < 0.01, Figure 3(c)). Further, we detected the death state of H9C2 cells after silencing TNNI3K and found that LPS aggravated H9C2 cell injury, while knocking out TNNI3K alleviated the cell injury induced by LPS (*P* < 0.01, Figure 3(d)). Meanwhile, TUNEL results indicated that si-TNNI3K-1 inhibited LPS-induced H9C2 cell apoptosis (*P* < 0.01, Figures 3(e) and 4).

### 3.4. Silencing TNNI3K Promoted Bcl-2 Expression and Inhibited Bax and Cleaved Caspased-3 Expression

We have shown that silencing TNNI3K could alleviate LPS-induced H9C2 cell apoptosis. To further explore the deep mechanism of TNNI3K affecting myocardial injury, we examined the expression of apoptosis-related proteins. As depicted in Figure 5(a), LPS significantly reduced Bcl-2 protein expression in H9C2 cells compared with the control group. On the contrary, the protein content of Bcl-2 increased evidently after cotransfection with si-TNNI3K (*P* < 0.01). In Figures 5(b) and 5(c), the results showed that LPS exposure significantly promoted the expression of Bax and cleaved caspased-3, while si-TNNI3K reversed the expression trend of the above proteins.

## 4. Discussion

SIMD is an important part of cardiovascular failure in septic shock, leading to high mortality and poor prognosis in patients with sepsis [2]. In this study, we presented the investigation of targeting TNNI3K for the treatment of SIMD in a rat septic model. Our silencing TNNI3K alleviated LPS-induced H9C2 cell injury by regulating apoptosis-related proteins.

LPS is the main component of gram-negative bacilli cell wall, evoking SIMD and organ injury [18]. Studies have shown that LPS-induced SIMD has been widely used in *in vitro* and *in vivo* model studies. For example, intraperitoneal injection of LPS can significantly increase the expression of inflammatory factors in myocardial tissue and cardiac dysfunction [19] and LPS can induce the production of inflammatory cytokines and reduce cardiac energy output [20]. In this study, we confirmed that LPS induced an increase in LDH release activity, CK activity, and apoptosis in rat cardiomyocytes, which is consistent with a previous study.

TNNI3K is a cardiomyocyte-specific kinase. A previous study has shown that in a TNNI3K overexpression knockout mouse model, TNNI3K can increase the area of ischemic heart infarction, induce mitochondrial ROS generation, and cause cardiomyocyte mitochondrial dysfunction and bioenergy damage [21]. TNNI3K is also associated with activation of p38 mitogen-activated protein kinase MAPK, which aggravates ischemic injury and cardiomyocyte death [22]. In this study, we found that the expression of TNNI3K was evidently increased in LPS-induced H9C2 cells, accompanied by significant damage to cardiomyocytes. Several studies on transgenic animals have strongly suggested that the activation of TNNI3K leads to a harmful phenotype. On the contrary, inhibiting its expression produces significant protection at baseline and postinjury [16, 23, 24]. Consistently, our results revealed that after silence TNNI3K, the LDH activity, CK activity, and apoptosis of H9C2 cells were significantly reduced, suggesting that TNNI3K plays an important role in regulating the progression of SIMD.

It has been reported that the occurrence of SIMD was closely related to apoptosis [25]. Bcl-2 is a family of evolutionarily related proteins, including both proapoptotic and antiapoptotic proteins. Among them, Bax is a proapoptotic gene, which releases proapoptotic substances into the cytoplasm to play a proapoptotic role. In contrast, Bcl-2 is an antiapoptotic gene that inhibits apoptosis by blocking oligomerization of proapoptotic proteins [26]. Caspase family proteins are one of the main executors of apoptosis, while caspase-3 was considered to be the most important terminal splicing enzyme in the process of apoptosis [27]. In our study, silencing TNNI3K inhibited the protein expression of Bax and cleaved caspased-3 and on the contrary increased the protein expression of Bcl-2, which was consistent with the results of TUNEL, indicating that si-TNNI3K could alleviate cell injury.

## 5. Conclusion

In this study, we mainly explored the functionality of TNNI3K and its potential molecular mechanisms in SIMD. We found that TNNI3K was upregulated in LPS-induced H9C2 cell and silencing TNNI3K alleviated LPS-induced H9C2 cell injury by regulating apoptosis-related proteins. Collectively, these observations indicated that TNNI3K may be utilized as a novel target to treat SIMD (Figure 6).

## Figures and Tables

**Figure 1:** TNNI3K was high expressed in LPS-induced H9C2 cells. (a) The mRNA level of TNNI3K in control group and LPS group. (b) The protein level of TNNI3K in the control group and LPS group. ∗ indicates comparison with the control group. LPS: lipopolysaccharide; TNNI3K: troponin I-interacting kinase.

**Figure 2:** LPS-induced myocardial injury. (a) The activity of creatine kinase in the control group and LPS group. (b) The LDH release activity in the control group and LPS group. (c) The mean fluorescence intensity of TUNEL staining. (d) TUNEL assay was conducted to detect the apoptosis of H9C2 cells. ∗ indicates comparison with the control group. LPS: lipopolysaccharide; LDH: lactate dehydrogenase.

**Figure 3:** Silencing TNNI3K alleviated LPS-induced H9C2 cell injury. (a) After knockout TNNI3K, the mRNA expression of TNNI3K in H9C2 cells was determined by qRT-PCR. (b) After knockout TNNI3K, the protein expression of TNNI3K in H9C2 cells was determined by western blot. (c) The activity of creatine kinase in different was detected by ELISA. (d) The LDH release activity in different was detected by LDH assay. (e) The mean fluorescence intensity of TUNEL staining in different groups. ∗ indicates comparison with the control group; # indicates comparison with the LPS group; & indicates comparison with the si-TNNI3K-1 group.

**Figure 4:** TUNEL assay was used to detect the apoptosis of H9C2 cells in different groups.

**Figure 5:** Silencing TNNI3K promoted Bcl-2 expression and inhibited Bax and cleaved caspased-3 expression. (a) The protein expression of Bcl-2 in different groups. (b) The protein expression of Bax in different groups. (c) The protein expression of cleaved caspase-3 in different groups. ∗ indicates comparison with the control group; # indicates comparison with the LPS group; & indicates comparison with the si-TNNI3K-1 group.

**Figure 6:** The diagram of molecular mechanism.

## Data Availability

The data used to support the findings of this study are available from the corresponding author upon request.
